# Discovering Knee Osteoarthritis Imaging Features for Diagnosis and Prognosis: Review of Manual Imaging Grading and Machine Learning Approaches

This article has been retracted.

**DOI:** 10.1155/2022/4138666

**Published:** 2022-02-18

**Authors:** Yun Xin Teoh, Khin Wee Lai, Juliana Usman, Siew Li Goh, Hamidreza Mohafez, Khairunnisa Hasikin, Pengjiang Qian, Yizhang Jiang, Yuanpeng Zhang, Samiappan Dhanalakshmi

**Affiliations:** ^1^Department of Biomedical Engineering, Universiti Malaya, 50603 Kuala Lumpur, Malaysia; ^2^Faculty of Medicine, Universiti Malaya, 50603 Kuala Lumpur, Malaysia; ^3^School of Artificial Intelligence and Computer Sciences, Jiangnan University, Wuxi 214122, China; ^4^Department of Medical Informatics of Medical (Nursing) School, Nantong University, Nantong 226001, China; ^5^Department of Electronics and Communication Engineering, SRM Institute of Science and Technology, Kattankulathur 603203, India

## Abstract

Knee osteoarthritis (OA) is a deliberating joint disorder characterized by cartilage loss that can be captured by imaging modalities and translated into imaging features. Observing imaging features is a well-known objective assessment for knee OA disorder. However, the variety of imaging features is rarely discussed. This study reviews knee OA imaging features with respect to different imaging modalities for traditional OA diagnosis and updates recent image-based machine learning approaches for knee OA diagnosis and prognosis. Although most studies recognized X-ray as standard imaging option for knee OA diagnosis, the imaging features are limited to bony changes and less sensitive to short-term OA changes. Researchers have recommended the usage of MRI to study the hidden OA-related radiomic features in soft tissues and bony structures. Furthermore, ultrasound imaging features should be explored to make it more feasible for point-of-care diagnosis. Traditional knee OA diagnosis mainly relies on manual interpretation of medical images based on the Kellgren–Lawrence (KL) grading scheme, but this approach is consistently prone to human resource and time constraints and less effective for OA prevention. Recent studies revealed the capability of machine learning approaches in automating knee OA diagnosis and prognosis, through three major tasks: knee joint localization (detection and segmentation), classification of OA severity, and prediction of disease progression. AI-aided diagnostic models improved the quality of knee OA diagnosis significantly in terms of time taken, reproducibility, and accuracy. Prognostic ability was demonstrated by several prediction models in terms of estimating possible OA onset, OA deterioration, progressive pain, progressive structural change, progressive structural change with pain, and time to total knee replacement (TKR) incidence. Despite research gaps, machine learning techniques still manifest huge potential to work on demanding tasks such as early knee OA detection and estimation of future disease events, as well as fundamental tasks such as discovering the new imaging features and establishment of novel OA status measure. Continuous machine learning model enhancement may favour the discovery of new OA treatment in future.

## 1. Introduction

Osteoarthritis (OA) is a degenerative joint disorder, characterized by cell stress and cartilage extracellular matrix degradation due to maladaptive repair responses actuated by micro- and macro-trauma [1]. Among the major weight-bearing joints, knee joint that comprises three compartments (medial tibiofemoral, lateral tibiofemoral, and patellofemoral) is most frequently affected by OA. The global prevalence of knee OA is 16% in the population aged 15 and above where the elders are the most affected subpopulation [2]. Primary knee OA occurs in elders due to wear and tear of cartilage tissues. However, younger individuals could develop secondary knee OA as a result of joint overuse or trauma.

The risk factors for knee OA include age, gender, obesity, injury, joint abnormalities, diet, excessive physical activity, physical inactivity, and genetic factors. People with symptomatic knee OA will suffer from debilitating knee pain, joint stiffness, joint swelling, physical disability, and difficulty in conducting activities of daily living (ADLs) [3]. Those symptoms are presented in a heterogeneous pattern, indicating that knee OA is a whole joint disorder instead of simple cartilage problem. The uptrend of knee OA prevalence is forecast due to increasing life expectancy and the rise of risk factors, such as obesity and ageing. It will gradually add burden to the healthcare resources, giving rise to a major economic burden in societies. Thus, action must be taken to relieve this future burden.

Knee OA disease management consists of two key elements: diagnosis and treatment. Both diagnosis and treatment work conjunctly to provide optimal disease management outcomes. The diagnosis identifies the existence of disease in patient itself based on signs and symptoms, whereas treatment works specifically to deal with the disease to trigger curative and palliative effects. The goal of treatment is to delay disease progression and to avoid the worst disease stage. The diagnosis can be done at multiple time points to monitor disease progression. By extending the fundamental knowledge of disease progression, the prognosis could be performed to predict future disease events and future treatment outcomes [4]. Currently, the unknown correlation between covariates has made knee OA prognosis remains unpractical. Medical experts hardly predict the right disease progression to formulate plan for disease prevention. To the best of our knowledge, there is no prognostic tool available in clinical practice. Recently, diagnostic and prognostic prediction models are conceptualized for the healthcare industry [4], and this idea could be adapted to upgrade the current knee OA management system.

Current knee OA diagnosis is mainly based on patient-reported outcome measures (PROMs) and X-ray imaging. Alternative knee OA diagnostic methods include physical assessment, arthroscopic assessment, joint aspiration, and advanced imaging systems. Knee OA diagnosis typically happens during moderate-to-late stage of disease, at a point where the irreversible joint damage is in evidence. It is worth noting that all currently available diagnostic methods require commitment from medical experts for high-level interpretation, which is usually time-consuming. To leverage current diagnostic systems, sensor technologies and machine learning algorithms are introduced, as inspired by the success of data-driven model in other healthcare departments [5–8].

Knee OA patients demand long-term disease management to control disease symptoms and to prevent disease complications. The OA continuum is presented in Figure 1, where the detection and intervention options over the entire OA evolution are illustrated. In most late OA scenarios, patients end up with knee arthroplasty [9], which is strongly undesirable. Several nonsurgical treatments are recommended at early-to-moderate OA stage to delay disease progression. Hitherto, there is no treatment approved by regulatory agencies to cure knee OA disease. Currently available medications are limited to symptoms relief. Most medications are still in clinical trial phase and lack supporting shreds of evidence to be commercially available. Among the developing OA treatments, intra-articular injection is prominent due to its promising pain relief effects on mid-to-late OA patients.

Researchers also suggested that the early detection of knee OA could be an effective strategy for OA disease management [10–12]. Presymptomatic detection allows the implementation of timely intervention, which can prevent further disease events such as cartilage degradation and bone damage. Additionally, there is evidence reporting that pre-osteoarthritis [13] could be a reversible process [14]. However, at early stage of knee OA, patients could be asymptomatic and the pathological changes are very subtle. Medical experts might misdiagnose the disease, causing patients to miss the best treatment time and subsequently develop permanent disability. To overcome this problem, high-end diagnostic system for early detection is strongly desired.

Recently, wearable sensors and wireless body area networks (WBANs) have been extensively studied for gait analysis and remote body condition monitoring [15, 16]. A framework namely artificial intelligence-based body sensor network framework (AIBSNF) [15] has been proposed to strategize the usage of body sensor networks (BSNs). The proposed framework optimizes real-time location system (RTLS) and wearable biosensors to gather multivariate, low-noise, and high-fidelity data. By analysing those data, the potential OA-related changes could be recognized. Besides, the quantification of varus thrust in patients with medial knee OA could be done with the placement of inertial sensor at mid-thigh [17]. Those findings reveal the potential of WBAN as an evaluation tool for rehabilitation performances and therapeutic effects. Although the findings are exciting and inspirational, however, the outcome domain for this data collection approach has not been established and has not been validated with clinical presentation.

The current knee OA management system is empowered with the emergence of data collection equipment, favouring data-driven studies for personalized medicine. Despite advancement in medical device and sensor technologies, the outcome measures of knee OA still demonstrate the lack of valid clinical reasoning. Medical experts scarcely find the right intervention for the right patient at the right time to sustain the knee OA disease. Most of the time, medical experts prescribe intervention by trial and error, until seeing the one works well for the patient. This healthcare approach is cost- and time-consuming, which is not ideal for large-scale knee OA management. Imaging features are one of the fast-growing outcome measures for objective OA assessment. This has motivated us to review the roles of knee OA imaging features in traditional and recent OA diagnosis and prognosis. We hope that this review study can provide insight into researchers regarding the emerging role of imaging features in AI-assisted diagnostic and prognostic models. The overview of this review study is illustrated in Figure 2.

## 2. Knee OA Imaging Features

Imaging modalities enable the visualization of knee joint structures, resulting in the production of digital images. The images are viewed by medical experts for manual knee image interpretation. The core of manual knee image analysis is the inspection of structural and pathological deviations as illustrated in Figure 3. Those deviations are usually examined carefully through qualitative visual judgements. Qualitative visual judgements are basically the spotted radiological findings, also known as imaging features, as described in Table 1. There are two things to be considered while observing knee OA imaging features, which are imaging modality and grading system. Understanding the basics of each imaging modality could give us the idea of which type of imaging features could be expected, whereas understanding the grading system could give us the clue of how to classify the disease severity using the known imaging features.

### 2.1. Knee Imaging Modalities

The existing knee imaging modalities include conventional radiography, magnetic resonance imaging (MRI), computed tomography (CT), nuclear medicine bone scan, ultrasonography, and optical coherence tomography (OCT). Among the imaging modalities, radiography is the most well-recognized OA diagnosis approach and is always used as standard diagnostic approach. MRI, CT, nuclear medicine bone scan, and ultrasonography are regarded as advanced imaging techniques, which are not routinely used in clinical practice. OCT imaging is still in the developmental phase for OA diagnosis. It is worth mentioning that OCT has demonstrated superior articular cartilage assessment. The characteristics of all imaging modalities are summarized in Table 2.

#### 2.1.1. Radiography

Radiography, which is also known as X-ray or roentgenography, is the gold standard for diagnosing OA. During X-ray imaging, radiation is passed through body. Calcium in bones will absorb the radiation, causing the bone structures to appear in white. The patient can be scanned in different positions, including supine, sitting, standing, fully extended, semiflexed, non-weight-bearing, and weight-bearing conditions. Weight-bearing condition is relevant to clinical assessment as the knee is usually under natural load when executing its functions. In addition, the Rosenberg view, a posteroanterior weight-bearing radiograph where the patient's knee is positioned in 45° of flexion, is more sensitive for JSN detection.

#### 2.1.2. Magnetic Resonance Imaging (MRI)

Magnetic resonance imaging (MRI) is an emerging imaging technique that works according to the theory of magnetic wave. During MRI scanning, the patient is positioned in supine position and sliding into a MRI tube. MRI technique has attracted the interest of many researchers due to its promising longitudinal and cross-sectional imaging outcomes.

#### 2.1.3. Computed Tomography (CT)

Computed tomography (CT) is an imaging modality that consists of rotating X-ray machines and computers to create images of internal body. CT scan can be done in both weight-bearing and non-weight-bearing conditions. When the evaluation of menisci and anterior cruciate ligament (ACL) is needed for clinical decision, CT arthrography will be performed [22]. Contrast dye will be injected before CT scan, to enable better visualization of targeted areas.

#### 2.1.4. Nuclear Medicine Bone Scan

Nuclear medicine bone scan is also known as bone scintigraphy. It is an imaging technique that utilizes the injection of radioactive tracer into patient's vein. Bone scintigraphy can help physicians to differentiate OA from other bone problems such as bone metastases and osteomyelitis. It should be noted that the detection of knee OA is not the main interest of nuclear medicine bone scan. This imaging technique will be used when medical expert suspects metabolic abnormalities at knee joint.

#### 2.1.5. Ultrasonography

Ultrasonography or ultrasound scanning is an imaging technique that utilizes ultrasound waves to assess soft tissues and joint structures. During the ultrasound scanning, the patient is positioned in supine condition with fully extended knees. The knee scanning is manually performed by physician in coronal plane by moving the scanner in the longitudinal direction. An ultrasound scanner is usually available at clinics for quick knee imaging assessment. Recently, a handheld wireless ultrasound device, namely the Clarius HD scanner, is developed and launched onto market. The real-time scanned image can be assessed directly on tablet or mobile phone, demonstrating great potential for point-of-care diagnosis.

#### 2.1.6. Optical Coherence Tomography (OCT)

Optical coherence tomography (OCT) is an intra-articular imaging technique featured with microscopic resolution for the detection of subtle degenerative changes in cartilage [13]. It is usually coupled with mechanical indentation to assess the anisotropy of cartilage under induced impact. Currently, OCT is used as a translational research tool to facilitate the clinical interpretation of quantitative MRI technologies for noninvasive articular cartilage assessment. OCT studies typically involve small size of animal samples. Although there are some studies that work on human samples, the experiment was done in ex vivo setting.

### 2.2. Knee OA Grading Systems

Radiographic findings and imaging features from each imaging modality are stratified onto an ordinal scale to form OA-specific grading system. The establishment of grading system has enabled the grading of disease severity, contributing to the foundation of knee OA diagnosis. The grading system not only allows qualitative assessment, but also enables semiquantitative assessment of OA disease. All currently available grading systems are summarized in Table 3. The Kellgren–Lawrence (KL) grading scheme derived from X-ray imaging features is commonly used as a standard for knee OA severity grading. Some grading systems such as OsteoArthritis Computed Tomography (OACT) are established and validated with the KL grading scheme.

### 2.3. Potentials and Limitations

Currently available imaging modalities manage to provide high-quality images to medical experts for OA diagnosis. Medical experts could inspect the imaging features using bare eyes and then interpret accordingly. They could also validate the diagnosis internally and externally based on their knowledge. This manual diagnostic approach has achieved satisfactory results in hospitals and clinics. Nonetheless, the reliability of human eyes is debatable as bias may occur due to fatigue, experience, and other personal factors. Kose et al. [23] pointed out that manual imaging diagnosis is greatly subjected to both interobserver variability and intraobserver variability, leading to inconsistent classification and poor result reproducibility.

Most established knee OA grading systems are derived from imaging features with respect to each imaging modality. The grading systems are composed of descriptive information and have guided medical experts in estimating OA severity. However, the grading schemes lack correlation with quantitative imaging measurements. The JSN percentage as described in radiographic grading schemes is difficult to be estimated through visual inspection. Moreover, the minimal JSN could be missed from detection. Presymptomatic knee OA diagnosis also remains a big challenge as the radiographic pattern at early OA is insignificant and unnoticeable. Researchers have previously suggested a few advanced quantitative examination approaches, work by extracting diagnostic meaningful structural details [24], such as joint space width [25, 26], cartilage thickness [27, 28], meniscal thickness [29], and tibiofemoral angle [30], from various images. Although the proposed methods have demonstrated the quantification of joint structures correlated with osteoarthritic joint, the diagnostic precision is not validated. Another observable limitation is the proposed workflow that lacks standard image calibration to ensure reproducibility. Despite the availability of preliminary application, quantitative assessment is not yet ready to be used independently for OA diagnosis. However, the quality of this assessment is appreciated and it can be used as ancillary information to aid the decision-making.

The image characteristics of each imaging modality are different due to the difference in theories. X-ray imaging is superior in terms of bony structure imaging, whereas MRI is superior in terms of soft tissue imaging. OA is a musculoskeletal disorder, where the evaluation of bony and soft tissue changes is equivalently important. It would be costly if a patient was subjected to multiple imaging techniques for a thorough diagnosis. Hence, researchers worked intensively on exploring hybrid imaging techniques that could combine the pros of different imaging systems [31–33].

From a research perspective, images from all imaging modalities can be stored and manipulated for further study, for instance, data mining or machine learning-related studies. The accumulation of data favours the development of an effective machine learning model. Worth noting, machine perception is superior to human perception in terms of time taken and reproducibility. Nevertheless, attention must be paid to apprehend the differences between human perception and machine perception in analysing the given input data or images.

## 3. Machine Learning for Image-Based Knee OA Diagnosis and Prognosis

Artificial intelligence (AI) is emerging in healthcare industry [34–36]. The innovation of AI in the medical field is the creation of a smart approach to gather patient insights for automated disease detection and predictive analysis. AI solution has been heavily studied for OA diagnosis [37, 38], and the outcomes are encouraging. Recently, OA prognosis has been an arising interest, which focuses on OA prevention. However, its implementation is greatly dependent on the shreds of evidence from OA disease progression monitoring. Most machine learning-related studies focused on imaging data, particularly X-ray and MRI images. Despite limited research quantity, a machine learning model was also applied on ultrasound images. The three major tasks in automated OA diagnosis are localization of knee joint (detection and segmentation), classification of knee OA severity, and prediction of knee OA disease progression. Some studies suggested that the model for the prediction of knee OA disease progression may be useful for prognosis [39]. The machine learning techniques for each task are summarized in Table 4.

### 3.1. Localization of Knee Joint

At the early stage of knee OA machine learning model, knee joint would be localized by object detection and segmentation approaches. Object detection involves the usage of a rectangular bounding box to localize region of interest, whereas object segmentation is a finer localization approach that involves the usage of a mask to lie on area of interest with an exact outline being drawn on the boundary of object. There are three different approaches being tried in previous studies, videlicet, pure object detection, pure object segmentation, and detection-segmentation combination. In detection-segmentation localization approach, knee joint is first detected, followed by the segmentation of its components such as meniscus, cartilage, and bones [76]. Object localization is an essential step that helps to extract the desired image segments and remove unimportant image parts, to ease the following machine learning operations.

#### 3.1.1. Detection of Knee Joint

A two-block knee joint localization method was proposed by Tiulpin et al. [43]. The first block was knee-anatomically based joint area proposal, whereas the second block was proposal scoring by histogram of oriented gradient (HOG) and the pretrained support vector machine classifier. This method could automatically annotate conventional knee radiographs within 14 to16 milliseconds, as well as high-resolution radiographs within 170 milliseconds with a sophisticated computer.

A pixel density-based approach that recognized large radiographic pixel values as bone image pixels was applied to detect and extract the desired cartilage region [41, 42]. Firstly, the computation was done using the HOG method and local binary pattern (LBP). Next, a decision tree classifier was used to classify the computed features. This approach achieved 97.86% and 97.61% accuracies with regard to the views of first and second medical experts [41]. After the cartilage detection, the resultant images were fed into an active contour algorithm to proceed with the segmentation process [42].

Tibiofemoral joint was detected by Mahum et al. [40] using matching technique with the knee image database. HOG was used to compute the similarity among the image blocks pixel by pixel, where the pixels with maximum similarity were chosen as region of interest.

Patellofemoral joint was detected by Bayramoglu et al. [44] from knee X-ray images. First, the detection of patella was performed using BoneFinder® software that works based on the random forest regression voting approach. Next, three regions of interest, namely inferior patellar region, superior patellar region, and whole patellar region, were localized. The local representation of textures in each ROI was captured by LBP.

A fully convolutional neural network (FCN) was used for automatic detection and extraction of knee joints in X-ray images [45, 46]. In this approach, a simple contour detection was performed based on the prediction outcomes from FCN. The maximum accuracy of automatic knee joint detection was 91.4% with the Jaccard index above 0.75. The slight error might be due to the variations in knee joint anatomy.

YOLOv2 network was utilized by Chen et al. [46] for knee joint detection in X-ray images. The process took only 10.5 milliseconds, which is relatively fast compared with other studies. The knee joint detection gained 0.858 mean Jaccard index and 92.2% recalling rate under 0.75 Jaccard index threshold.

#### 3.1.2. Segmentation of Knee Joint Components

Knee cartilage segmentation was performed by Faisal et al. [28] on ultrasound images using locally statistical level set method (LSLSM). The authors compared the proposed method with local Gaussian distribution fitting (LGDF) and locally weighted K-means variational level set (WKVLS) methods, whereas manual segmentation was served as ground truth data. LSLSM outperformed LGDF and WKVLS with mean dice coefficient (DC) of 0.91 ± 0.01. Nonetheless, LSLSM still exhibited limitation where it required connected-component labelling to post-process the segmented images. Similar work was done by Desai and Hacihaliloglu [27] using a local-phase-based image processing approach. Seed was initialized at localized bone surfaces to guide the segmentation. Three segmentation methods, namely random walker, watershed, and graph cut, were studied. The random walker method demonstrated the best segmentation performance among the evaluated models with DC of 0.90. This study was limited to 2D ultrasound image segmentation. It should be noted that ultrasound images are prone to speckle noise [77], and hence, careful image preprocessing is required.

To segment subchondral bone, Gandhamal et al. [48] proposed a three-phase fully automated segmentation method. It was initiated by a preprocessing phase, where the MRI contrast enhancement was done with a gray-level S-curve transformation, before proceeding to the automatic seed point detection utilizing a three-dimensional multi-edge overlapping method. Bone region extraction was then executed with distance-regularized level set (DRLS) evolution. Lastly, it was subjected to the post-processing phase, which involved the identification, correction, and smoothing of leakages along the bone boundary regions with a boundary displacement technique. The sensitivity, specificity, and DC were above 90% for the segmentation of femoral and tibial bones, indicating good overall segmentation performance. However, the small bone might be missed from being segmented due to the threshold limit.

Chang et al. [57] segmented subchondral bone and cartilage using U-Net. The authors also developed a new bone-shaped measure called subchondral bone length (SBL) that can be made on segmented images. SBL characterizes the degree of overlying cartilage and bone flattening. The study revealed that the change in SBL from baseline is proportional to the extent of pain and disability.

In terms of MRI cartilage and meniscal segmentation, a study was carried out to compare the performance between manual approach and U-Net [29]. Based on the findings, U-Net was comparable to manual segmentation with promising efficacy and precision. This was agreed by another study where the automatic segmentation of cartilage and meniscus was done using 2D U-Net in 8 seconds before feeding into a classification model [56]. A similar approach was employed by Norman et al. [55] on bilateral X-ray images to localize the knee joint in 1.49 second.

Cheung et al. [49] have tested the segmentation ability of four models, namely CUMed-Vision, U-Net, DeepLabv3, and Res-U-Net. All four models were used to segment distal femur and proximal tibia. Res-U-Net gave the best segmentation outcome with the highest mean intersection over union score at 0.989. In addition, Res-U-Net demonstrated less validation loss as compared to other tested models.

A real-time femoral condyle cartilage tracking algorithm, known as Siam-U-Net, was proposed by Dunnhofer et al. [50]. Siam-U-Net is a combination of the Siamese tracking model and U-Net. In this combined model, the femoral condyle cartilage was segmented for tracking purpose. The model was validated against two video object segmentation methods, which were one-shot video object segmentation (OSVOS) and reference-guided mask propagation (RGMP). Siam-U-Net outperformed the two validated models with the best segmentation result at DC of 0.70 ± 0.16 in executing temporal tracking. In terms of spatiotemporal tracking, the model performed slightly better with DC of 0.71 ± 0.16. Even so, this study reported high intraoperator variability, implying the operational uncertainty of application.

Ten encoder-decoder-based CNN architectures, including U-Net Vanilla, FC-DenseNet-56, FC-DensetNet-67, FC-DenseNet-103, LinkNet-34, TernausNet-11, TernausNet-16, AlbuNet, Attention U-Net, and LadderNet, were compared by Yong et al. [47]. Those architectures were used to perform the knee cartilage segmentation on MRI images. Based on the results, U-Net Vanilla gave the best segmentation outcomes. Interestingly, LadderNet provided comparable results using the least trainable parameters. This architecture could be an alternative option when the computational resources are limited.

Liu [51] applied cycle‐consistent generative adversarial network (CycleGAN) onto two types of MRI images, namely fat‐suppressed T2‐weighted fast spin‐echo (T2‐FSE) and proton density‐weighted fast spin‐echo (PD‐FSE), to segment the desired knee bones and cartilages. In this study, the standard U‐Net structure was modified into a new version called R-Net, which could produce dual outputs. The accuracies of bone segmentation were 0.94 to 0.96 and 0.93 to 0.95 DC for femur and tibia, respectively, whereas the cartilage segmentation accuracies were 0.59 mm to 0.84 mm and 0.70 mm to 0.71 mm average symmetric surface distance (ASSD) for femoral and tibial cartilages. The obtained results were comparable to U-Net, meanwhile outperformed multi-atlas registration and direct registration methods. The findings were consistent with the study under Kessler et al. [52], who has investigated the use of conditional generative adversarial networks (cGANs) for automated semantic segmentation of MRI knee bones, cartilage, and muscle tissues.

3D fully connected conditional random field (FC-CRF) and 3D simplex deformable modelling were incorporated into a convolutional encoder-decoder (CED) knee joint segmentation model by Zhou et al. [53]. Excellent performance with mean DC over 0.9 was reached in the segmentation of femoral bones, tibial bones, muscles, and other nonspecified tissues. The DC of femoral, tibial, and patellar cartilages and patella, meniscus, patellar tendon and quadriceps, and infrapatellar fat pad lay between 0.8 and 0.9. In this study, the model was only evaluated on 3D-FSE images. It should be noted that the training of CED network required the expense of huge computational resources. Meanwhile, a large amount of pixel-wise annotated training data was needed for the evaluation of each new tissue contrast.

3D segmentation was performed by Huang et al. [54] to extract tibial and femoral cartilages. MRI images are processed in a four-step approach, starting from 2D segmentation by cascaded U-Net models and meshing with marching cubes, followed by 3D thickness map computation, image registration using atlas image, and lastly 3D thickness map projection. It is worth noting that 3D segmentation of cartilage is crucial for whole knee joint reconstruction. Liukkonen et al. [58] have attempted to simulate cartilage degeneration on reconstructed 3D knee joint model. The cartilage degeneration simulation has shown promising result in discriminating knee OA progression at 4-year follow-up.

### 3.2. Classification of Knee OA Severity

The identification of knee OA severity is a main diagnostic task. Most studies built the classification model based upon the KL grading system [45, 46, 55, 60, 62]. A few studies focused on the classification of osteoarthritic knee [59], or osteoarthritic meniscus and cartilage tissue [56].

Hirvasniemi et al. [59] utilized MRI tibial radiomic features to build an elastic net model that could discriminate osteoarthritic knee. The proposed model obtained an AUC of 0.80 and outperformed the covariate model with an AUC of 0.68. The authors strongly recommend the usage of radiomic features for the classification of OA incidence.

Pedoia et al. [56] employed a 3D convolutional neural network (CNN) and a random forest classifier to execute a three-class classification of meniscal lesion on MRI data. The optimal performances, indicated by accuracies of 80.74%, 78.02%, and 75.00% with respect to normal, small, and complex large lesions, were yielded by considering the demographic factors. Although the model performed fairly well, the model pitfall was indicated. The model demonstrated decreasing performance in grading higher degree of meniscal damage, implying that the model's generalizability could be disturbed by the structural irregularities in a certain pattern.

Tiulpin et al. [60] utilized a deep Siamese CNN model to automatically grade the knee OA severity in the X-ray images based on KL classification. A quadratic Kappa coefficient of 0.83 and average multiclass accuracy of 66.71% were achieved after making comparison with the annotations provided by a committee of medical experts. In addition, an AUC of 0.93 was reported. Notably, this model was well-performed from clinical perspective as it managed to produce better classification outcome for early OA cases compared with other models.

Mahum et al. [40] used hybrid feature descriptors, CNN with HOG, and CNN with LBP to extract meaningful features from radiographs. Three classifiers, support vector machine, random forest, and K nearest neighbour, were employed and compared. CNN with HOG coupled with K-nearest neighbour classifier produced the best accuracy at 97.14% for all KL grades.

Bayramoglu et al. [44] exemplified automated diagnosis of patellofemoral OA using gradient boosting machine (GBM) and deep CNN. The authors trained the GBM model to identify radiographic patellofemoral OA from handcrafted texture features. Deep CNN worked directly on ROI without texture descriptor. The proposed method produced optimal classification results with 0.889 AUC, and Chen et al. [46] incorporated a novel adjustable ordinal loss into four deep CNNs, which were ResNet, VGG, DenseNet, and InceptionV3, to classify knee OA KL grade based on X-ray images. Among the four tested models, VGG-19 with proposed ordinal loss attained the best performance with average multiple-class accuracy of 67.70% and mean absolute error (MAE) of 0.344. Further study was conducted by Yong et al. [61] by adopting ordinal regression module with cumulative link loss function into six neural network architectures, namely VGG, GooLeNet, ResNet, DenseNet, ResNeXt, and MobileNetV2. KL grades of 0, 2, 3, and 4 were correctly identified at rate of 70% and above, whereas KL grade 1 classification showed relatively poor performance at 38.51%. However, this approach still demonstrated improvement in terms of KL grade 1 classification when compared to baseline approach and Chen et al. [46]. Both studies reported that the misclassification rate could be reduced by ordinal regression module and better classification outcomes were yielded.

Abedin et al. [45] have developed four prediction models, which were a CNN model that was trained with X-ray images, linear mixed-effects models, elastic net, and random forest models that were fed with clinical data. The prediction results showed that elastic net and linear mixed-effects models outperformed CNN and random forest.

In knee X-ray data, geometric distortions were often found on cartilage region, which could lead to misrepresentation. Yet, those distorted images might contain underlying information indicating knee OA progression. The extraction of significant regions from distorted images is a difficult task. To address the issue, Gornale et al. [42] has proposed Hu's invariant moments, which were computed from the segmented region to enhance the classification performance. Using a K nearest neighbour classifier, 99.80% and 98.65% accuracies were attained in accordance with opinions of first and second medical experts.

Several studies have demonstrated the use of DenseNet for the automatic radiographic KL classification [55, 62]. The DenseNet model in the study conducted by Norman et al. [55] achieved testing sensitivity rates at 83.7%, 70.2%, 68.9%, and 86.0% and specificity rates at 86.1%, 83.8%, 97.1%, and 99.1%, for healthy, mild, moderate, and severe OA conditions, respectively. This was agreed by the DenseNet model developed by Thomas et al. [62], which obtained an average F1 score of 0.70 and an accuracy at 0.71 for the full test set with a total of 4090 subjects. Interestingly, the automated KL grading could be performed within 30 seconds using a single CPU, and within 2 seconds using a GPU [62], displaying a remarkable time-saving potential.

Tiulpin and Saarakkala [63] have demonstrated the ensemble method by utilizing two 50-layer deep neural networks, which were SE-ResNet-50 and SE-ResNet-50-32x4d. The model predicted a total of six knee joint radiographic features according to the OARSI grading atlas and predicting the KL grade.

### 3.3. Prediction of Knee OA Disease Progression

Prognosis or prediction of future knee OA disease event is a formidable hurdle in knee OA disease management. Previously, knee OA disease was modelled as a linear process, but this assumption was criticized by multiple researchers [78, 79]. Many longitudinal studies were carried out to model the knee OA disease progression [80]. Multiple time-point data on a pool of individual patients were collected to track the disease trajectory over a period of time [80]. The knee OA progression prediction model could help to distinguish individuals with high risk of rapid disease progression and predict the likeliness of patients to benefit from specific intervention [81].

Current state-of-art knee OA disease progression prediction models mainly perform binary classification to discriminate between progressors and nonprogressors [39, 64, 66]. Multiclass classification was developed with the expansion of progressors' groups [39, 65]. In addition, some studies focused on the prediction of total knee replacement (TKR) as future event [68, 75]. None of the knee OA assessment methods alone could provide highly comprehensive information to make robust predictions or prognoses. Hence, non-imaging data or covariates such as patient characteristics, comorbidities, medical history, anthropometric data, and lifestyle were included in most research projects.

Lazzarini et al. [64] have developed five 30-month knee OA incidence prediction models using ranked guided iterative feature elimination (RGIFE) approach and random forest algorithm. The two lowest performances were produced by JSN outcome measures with 0.731 and 0.737 area under curves (AUCs) for lateral and medial compartments, respectively. Yet, the authors believed that the performances were still fair enough. The study also affirmed that the KL incidence OA outcome measure could be an influential input variable to the prediction model with 0.823 AUC full. It should be noted that this study was limited to the population of middle-aged overweight and obese women.

Ntakolia et al. [66] extracted a total of 725 features from nine categories, where only 21 features were under medical imaging outcome category, to build a prediction model specifically for medial JSN progression using clustering, feature engineering, and classification algorithms. It revealed that bounding the JSN progression of both sides of knee could achieve the highest maximum prediction accuracy at 83.3% with the least feature usage at amount of 29, compared with bounding the JSN progression of individual knee, with the usage of logistic regression classifier. The right knee only achieved 77.7% maximum accuracy by feeding 88 features into the support vector machine model. Although the left knee achieved slightly better maximum accuracy at 78.3% using the logistic regression model, the feature amount was almost double of right knee at 164. In this proposed model, although the features from medical imaging outcome were used as main contributors, the importance of other features such as symptoms, anthropometric data, and medical history information was recognized. Non-imaging data were included to ensure feature heterogeneity.

Hafezi-Nejad et al. [67] applied multivariate logistic regression and multilayer perceptron (MLP) models onto MRI images to examine the role of cartilage volumes and the interval changes in the corresponding cartilage volumes, as well as the prediction with respect to medial compartment joint space loss progression. The results revealed that the cartilage volumes in the lateral femoral plate are predictive of medial joint space loss progression.

An attempt was made by Chan et al. [71] to build a knee OA onset and deterioration predictive model using MLP. 4,181 knees from Osteoarthritis Initiative were used. Six risk factor categories, namely living habits, demographic information, radiographic information, mechanical factors, metabolic syndromes, and symptomatic information, were included as input variables. Although this model has obtained acceptable results with AUC of 0.843 and 0.765 for knee OA onset and deterioration predictions, this model was not insufficiently validated.

Halilaj et al. [39] employed least absolute shrinkage and selection (LASSO) regression to construct a prognostic tool that could use one-year data to predict eight-year disease progression. The OA progression was categorized into “nonprogressing” and “progressing” based on JSN assessment and further classified into “worsening,” “stable,” and “improving” based on pain score. The authors found that radiographic progression could be predicted accurately with AUC of 0.86 utilizing data from two visits in a span of one year, whereas pain progression could be predicted accurately with AUC of 0.95 utilizing single-visit data. In addition, the findings indicated that there is no association between JSN and pain progression. However, this study only targeted US OA patients, and the model's generalizability should be tested.

Joint space width data were utilized by Cheung et al. [49] to feed into the XGBoost model for knee OA severity classification. The proposed 64-point multiple-joint space width data demonstrated moderate performance in estimating knee OA progression within 48 months, with 0.621 AUC, more superior than the frequently used minimum-joint space width data that only achieved 0.554 AUC. However, attention should be focused on the computational complexity in terms of time taken and memory requirements, which has not been mentioned by the authors.

Guan et al. [70] built three models, namely deep learning model using the X-ray images as input, artificial neural network model using the demographic and radiographic risk factors as input, and a combined joint training model, to predict the progression of radiographic joint space loss. In the combined joint training model, the deep learning network was used to extract information from baseline knee radiograph as a feature vector, which was further concatenated with the risk factor data vector. Based on the final results, the combined joint training model produced the best performance, followed by the deep learning model and artificial neural network model. This study was limited to 48-month follow-up period.

Prediction for pain progression from baseline X-ray images was accomplished by Guan et al. [74] using a deep learning approach. This application has gained AUC of 0.770. The performance was further enhanced and boosted to AUC of 0.807 with the inclusion of demographic and clinical data. Pierson et al. [73] have demonstrated the usage of X-ray images for pain prediction using CNN approach. This research has put attention on unravelling the pain disparities in underserved population. The proposed algorithmic pain prediction (ALG-P) accounted for 43% of racial pain disparity, outperforming the KL grading approach.

Tiulpin et al. [72] developed a multimodal machine learning model to predict the risk of knee OA progression. The risk of OA progression was divided into three states: no progression, rapid progression, and slow progression. Firstly, raw radiographic data were fed into a deep CNN model to estimate the probability of knee OA progression. The deep CNN model also predicted knee OA severity at current time point in terms of KL grades as an auxiliary outcome. The prognosis from deep CNN was improved by fusing its prediction with non-imaging data, such as baseline patient characteristics, clinical examination, and optional KL grade identified by a radiologist, using a GBM. This approach achieved 0.79 AUC and 0.68 average precision (AP) and performed better than the reference approach that was based on logistic regression, which only obtained 0.75 AUC and 0.62 AP.

Widera et al. [65] employed six machine learning algorithms and compared their respective knee OA progression prediction performances. The predicted classes were divided into nonprogressive, progressive pain, progressive structural change, and progressive structural change with pain. The results indicated that random forest was the best machine learning algorithm as its cost-sensitive learning outperformed the balanced learning on downsampled training set. The results were further improved with the duo classifier. It is important to note that this study only focused on a short progression time window based on the setting of clinical trials.

Huang et al. [54] attempted to quantify OA progression across time points and subjects. The authors proposed a dynamic functional mixed-effects model (DFMEM) to simultaneously discriminate individual abnormal regions on MRI images at baseline, 12 months, 24 months, and 48 months. The relationship between cartilage thickness and covariates of interest, which represents spatiotemporal heterogeneity, was captured by the model. This model is significant in discovering the cartilage change over certain period of time, to make a fundamental contribution to the understanding of OA disease.

The prediction of TKR was executed by Tolpadi et al. [68] using a deep learning pipeline made of DenseNet-121 and logistic regression. The efficiency of model was compared between the usage of X-ray and MR images as well as with and without non-imaging information. Although the integrated X-ray model (88.4 ± 0.094%) delivered higher accuracy than integrated MRI model (78.5 ± 0.134%), however, integrated MRI model (81.8 ± 0.643%) displayed better sensitivity over integrated X-ray model (66.3 ± 0.924%) across entire OA stages, particularly at no OA group (92.2 ± 1.68%). AUCs of MRI models outperformed X-ray models at no OA group. The integrated MRI model obtained AUC of 0.834 ± 0.036. Importantly, this model competently predicted TKR event among the patients without OA at baseline with AUC of 0.943 ± 0.057%.

Seven machine learning methods, namely Cox, DeepSurv, random forest, linear/kernel support vector machine, and linear/neural multitask logistic regression, were used by Jamshidi et al. [75] to build a prediction model to prophesy risk and time to TKR for an OA-affected knee. At the beginning of the study, ten most important features, including X-rays, MRI feature bone marrow lesions (BMLs) in medial condyle, hyaluronic acid injection, performance measure, medical history, and knee symptoms, were identified by Lasso's Cox among a total of 1107 features. The prognostic power of the ten selected features was then analysed by the Kaplan–Meier before feeding into the machine learning models. Based on the results, Cox, DeepSurv, and linear SVM models displayed the highest accuracy with C-index of 0.85, Brier score of 0.02, and AUC of 0.87. However, the authors have selected DeepSurv to build the prediction model for the estimation of time to TKR after considering the model's ability to perform nonlinear analysis. Interestingly, comparable prediction outcomes (C-index of 0.85, Brier score of 0.02, and AUC of 0.86) were yielded with the usage of only three features, specifically BML, KL grade, and knee symptoms.

Bowes et al. [69] developed a new measure for OA status based on MRI images, namely B score. B score indicates the distances along OA vector. OA vector was created from the mean shape of OA population at four time points, which were baseline, one year, two years, and four years. In large observational cohort, B score managed to generate logistic regression models for clinically important outcomes that ranged from pain, functional limitation, and TKR. The predictive validity of proposed approach was similar to those of the existing X-ray imaging standard.

## 4. Research Gaps and Future Prospects

This review study presents the utilization of imaging features in manual grading systems and machine learning models. It also discloses the existing roles of machine learning approach in image-based knee OA diagnosis and prognosis that range from knee joint localization, OA severity classification, and OA progression prediction. Additionally, this study points out the optimal diagnostic outcomes achieved by machine learning algorithms. Despite favourable indications, three research gaps are highlighted for discussion.

The first research gap is the knee OA disease trajectory; over time, it is still not fully understood. No research has been conducted to establish a baseline model that represents lifetime knee OA progression. The significance of baseline knee OA disease trajectory over time is to demystify the understanding of knee OA evolution. This knowledge could give insights into the detection of early OA and presymptomatic OA. It could be used as a baseline or default mode for machine learning model, so the disease could be suspected once the patient's input data exhibit a pattern deviation. In addition, morphologic changes in meniscus, cartilage, and bone due to OA should be explored at imaging level.

Secondly, knee OA is a heterogeneous and multifaceted disease. Apart from radiological signs, other non-imaging data such as demographic data, comorbidities, clinical factors, pain intensity, and gait performances are equally important. The non-imaging data should be used as variables for OA incidence detection. Ideally, in a data-driven diagnostic model, the more the OA symptoms and risk elements are included, the more robust the diagnostic outcome is. This could favour precision medicine in OA management [82]. Yet, big data storage is required for this implementation. Currently, the largest OA database is Osteoarthritis Initiative with the involvement of 4,796 participants, and data are still increasing. Researchers should focus on how to manipulate the massive data intelligently to produce optimal diagnostic and prognostic outcomes. The identification of useful risk factors and risk stratification should be a research intention.

Thirdly, there are no radiology-based monitoring systems for the evaluation of intervention effectiveness. Current medical practice in knee OA management focuses on diagnosis and treatment. However, only diagnosis mode is periodically validated with the evaluation of knee OA imaging features. As more intra-articular treatment, orthobiologics, and disease-modifying osteoarthritis drugs (DMOADs) are subjected to clinical trial phase, there is an increasing demand for continuous radiology-based observation of therapeutic effect. Thus, an automated knee condition monitoring model should be created as an assistive tool. Besides, when any treatment has been approved for routine use in hospital, a knee OA disease progression prediction model could facilitate the medical experts to make prescription wisely by predicting the probability of optimal intervention outcomes.

## 5. Conclusion

Imaging features are important elements for the identification of OA incidence. The grading of OA severity is accomplished by stratification of imaging features. Prognosis is an emerging disease management strategy for future medical practice. Its implementation could be realized with machine learning model. Based on previous studies, all machine learning models are relatively reliable. Automated knee joint detection and segmentation of knee joint components are significantly faster than manual detection and segmentation without compromising the high accuracy rate. The automated knee OA classification model has provided promising result, which is comparable to the medical experts' interpretation. Importantly, the classification outcome of proposed machine learning models tends to be more reproducible than the diagnosis of medical experts. Knee OA disease progression prediction model has demonstrated prognostic power in terms of estimating possible OA onset, deterioration, progressive pain, progressive structural change, progressive structural change with pain, and time to TKR incidence. The presented findings further convince the future prospects of machine learning techniques in early knee OA detection, estimation of future disease events, and discovery of new disease treatment. Nevertheless, future work should be focused on fundamental exploration of imaging features using machine learning approach, such as identifying pain-associated imaging features and investigating the imaging features indicating the improvement caused by knee OA intervention, to bridge the gap between diagnosis and intervention [83].

## Figures and Tables

**Figure 1:** Knee OA continuum in terms of detection and intervention.

**Figure 2:** Overview of this review study (“∗” indicates numbering of section where the topic will be discussed).

**Figure 3:** Illustration of knee OA features and pathologies with respect to healthy knee.

**Table 1:** Radiological OA features.

OA features	Description
Joint space narrowing (JSN) [18]	Usually asymmetric, commonly happens at medial tibiofemoral and patellofemoral compartments
Osteophyte formation [18]	Formation of bone spurs
Cyst/geode formation [18]	Formation of fluid-filled cavities when synovial fluid is forced into subchondral bone
Subchondral sclerosis [18]	Increased bone density or thickening of bone when bone grows in the area originally belongs to cartilage
Coronal tibiofemoral subluxation [18–21]	Misaligned joint surface, causing altered shape of femoral condyles and tibial plateau

**Table 2:** Imaging techniques for knee OA diagnosis.

Imaging technique	Working principle	Pros	Cons	Detectable OA features	Grading scale
X-ray imaging/radiography/roentgenography	Ionizing radiation from X-ray passes through patient's body in one direction	(i) Low cost	(i) Mostly limited to 2D visualization	(i) Joint space narrowing	(i) Kellgren–Lawrence (KL)
		(ii) Routine OA imaging in clinical practice	(ii) Less sensitive to change over time	(ii) Osteophyte formation	(ii) Ahlbäck
		(iii) Allows bony structure visualization	(iii) Lack of soft tissue visualization	(iii) Cyst formation	(iii) Brandt
		(iv) Subjects can be scanned in different positions, including supine, sitting, standing, fully extended, semiflexed, non-weight-bearing, and weight-bearing conditions	(iv) Prone to positioning errors	(iv) Subchondral sclerosis	(iv) Osteoarthritis Research Society International (OARSI)
			(v) Risk of radiation		(v) International Knee Documentation Committee (IKDC)
					(vi) Fair bank
					(vii) Jäger-Wirth

Magnetic resonance imaging (MRI)	Protons in patient's body are stimulated using magnetic fields	(i) Permits visualization of intra-articular structures and soft tissues	(i) Expensive	(i) Joint space narrowing	(i) Modified Outerbridge classification
		(ii) Permits visualization of cartilage biochemical properties and pathological features	(ii) Intolerable to metal implant	(ii) Bone marrow lesions	(ii) Whole-Organ MRI Scoring (WORMS)
		(iii) Allows 2D and 3D visualization	(iii) Risk of overdiagnosis		(iii) Knee Osteoarthritis Scoring System (KOSS)
					(iv) Boston Leeds Osteoarthritis Knee Score (BLOKS)
					(v) MRI Osteoarthritis Knee Score (MOAKS)

Computed tomography (CT)	Ionizing radiation is passed through patient's body using motorized X-ray source before reaching the electronic detector	(i) Permits visualization of bony structure and calcified tissue (e.g., intra-articular calcium crystal deposition)	(i) Expensive	(i) Osteophyte formation	(i) OsteoArthritis Computed Tomography (OACT)
		(ii) Allows study of osteoarthritic biomechanics using weight-bearing and kinematic four-dimensional CT	(ii) Risk of radiation	(ii) Cyst formation	
		(iii) Allows study of joint metabolism	(iii) Requires intra-articular injection of contrast material in the case of CT arthrography, may cause allergic reaction	(iii) Subchondral sclerosis	
		(iv) Potential image-guided therapy tools with CT arthrography			
		(v) Allows 2D (slices) and 3D visualization			

Nuclear medicine bone scan	Radioactive tracer is injected into patient's vein is absorbed by metabolically active cells and tissues	(i) Enables radiopharmaceutical localization	(i) Injection of radioactive tracer	(i) Osteophyte formation	Nil
		(ii) Allows evaluation of injury status	(ii) Complicated procedures	(ii) Cyst formation	
		(iii) Differentiation of OA from bone metastases and osteomyelitis	(iii) No grading system for OA disease severity	(iii) Subchondral sclerosis	
		(iv) 2D and 3D visualization		(iv) Bone marrow lesions	

Ultrasonography	Knee joint is scanned with sound waves	(i) Low cost	(i) Limited to 2D visualization	(i) Osteophyte formation	(i) Ultrasonographic grading scale
		(ii) Evaluation of ligaments and synovium	(ii) Poor contrast caused by fat and air		
		(iii) Real-time assessment	(iii) Limited to evaluation of the far inner margins of lateral and medial femorotibial joints		
		(iv) Portable	(iv) Risk of overdiagnosis		
		(v) Potential image-guided therapy tools			
		(vi) Better spatial resolution			

Optical coherence tomography (OCT)	Cartilage sample is scanned with infrared light	(i) Evaluation of articular cartilage at resolution up to micron scale at 4 to 20 *μ*m near real-time assessment	(i) Not applicable to in vivo assessment	(i) Cartilage surface roughness	(i) Degenerative joint disease (DJD) classification
		(ii) Portable	(ii) Time-consuming	(ii) Degeneration of articular cartilage	
		(iii) Potential image-guided therapy tools			
		(iv) 2D and 3D visualization			

**Table 3:** Summary of knee OA grading systems based on imaging modalities.

Imaging modalities	OA grading system	Examined OA features	Pros	Cons
X-ray images	KL	(i) Osteophyte	(i) Universally accepted knee OA grading system	(i) Overemphasizes the significance of osteophytes as compared to JSN
		(ii) JSN	(ii) Indicates OA changes in medial compartment better	(ii) Poor reliability for OA changes in lateral compartment
		(iii) Bone end deformity		(iii) Poor inter- and intraobserver reliabilities
		(iv) Subchondral sclerosis		
	Ahlbäck	(i) JSN	(i) Greater emphasis on JSN than osteophytes by assuming the joint space reduction as an indirect sign of cartilage loss	(i) Poor inter- and intraobserver reliabilities
		(ii) Bone attrition		
	Brandt	(i) Percentage of JSN	(i) Greater emphasis on JSN than osteophytes	(i) Poor inter- and intraobserver reliabilities
		(ii) JSN associated osteophytes	(ii) Good correlation with arthroscopic damage	
		(iii) JSN associated subchondral sclerosis		
		(iv) JSN associated subchondral cysts		
	OARSI	(i) Percentage of JSN	(i) Most widely used individual OA feature scale with example images	(i) Only focus on JSN feature
	IKDC	(i) Joint space width	(ii) Best combination of good interobserver reliability and medium correlation with arthroscopic findings	(i) Only focus on joint space width
	Fair bank	(i) Squaring of tibial margin	(i) Involves many radiographic features	(i) Limited to post-meniscectomy condition
		(ii) Flattening of femoral condyle		(ii) Lack of knowledge about its reliability
		(iii) Sclerosis of tibial margin		
		(iv) Hypertrophic changes		
		(v) JSN		
	Jäger-Wirth	(i) Osteophytes	(i) Involves many radiographic features.	(i) Lack of knowledge about its reliability
		(ii) JSN		
		(iii) Arthrosis		

MRI images	Modified Outerbridge classification	(i) Fat-saturated proton density sequences of chondromalacia patella and chondral surface	(i) Greater emphasis on cartilage morphology	(i) Require validation with arthroscopic examination
				(ii) No bony assessment
	WORMS	(i) Cartilage	(i) Greater emphasis on cartilage and bone morphologies	(i) Tedious interpretation task
		(ii) Bone marrow lesions		
		(iii) Subchondral cysts		
		(iv) Bone attrition		
		(v) Osteophytes		
		(vi) Effusion synovitis		
		(vii) Meniscal tears		
		(viii) Ligaments		
		(ix) Periarticular cysts		
		(x) Bursitis		
		(xi) Loose bodies		
	KOSS	(i) Cartilage	(i) Greater emphasis on cartilage and bone morphologies	(i) Tedious interpretation task
		(ii) Bone marrow lesions		
		(iii) Subchondral cysts		
		(iv) Osteophytes		
		(v) Effusion synovitis		
		(vi) Synovial thickening		
		(vii) Meniscal extrusion		
		(viii) Meniscal tears		
		(ix) Popliteal cysts		
	BLOKS	(i) Cartilage	(i) Greater emphasis on cartilage and bone morphologies	(i) Tedious interpretation task
		(ii) Bone marrow lesions		
		(iii) Osteophytes		
		(iv) Effusion synovitis		
		(v) Hoffa synovitis		
		(vi) Meniscal extrusion		
		(vii) Intrameniscal signal		
		(viii) Meniscal tears		
		(ix) Meniscal maceration		
		(x) Meniscal cyst		
		(xi) Ligaments		
		(xii) Periarticular cysts		
		(xiii) Bursitis		
		(xiv) Loose bodies		
	MOAKS	(i) Cartilage	(i) Greater emphasis on cartilage and bone morphologies	(i) Tedious interpretation task
		(ii) Bone marrow lesions	(ii) Cover most OA features	
		(iii) Osteophytes		
		(iv) Effusion synovitis		
		(v) Hoffa synovitis		
		(vi) Meniscal extrusion		
		(vii) Intrameniscal signal		
		(viii) Meniscal tears		
		(ix) Meniscal maceration		
		(x) Meniscal cyst		
		(xi) Hypertrophy		
		(xii) Ligaments		
		(xiii)Periarticular cysts		
		(xiv) Bursitis		
		(xv) Loose bodies		

CT images	OACT	(i) JSN	(i) Emphasis on two knee compartments: tibiofemoral and patellofemoral joints	(i) Lack of validation result
		(ii) Osteophytes		
		(iii) Cysts		
		(iv) Sclerosis		

Ultrasonography	Ultrasonographic grading scale	(i) Osteophytes	(i) Depends on the shape of distal femoral osteophytes	(i) Features may be distorted by noise
		(ii) Projection from femoral condyle		(ii) Limited to primary knee OA

OCT images	DJD classification	(i) Cartilage surface irregularities	(i) Deep examination of cartilage	(i) Difficult to collect samples
		(ii) Tissue disorganization in cartilage		(ii) Only focuses on cartilage changes
		(iii) Fibrocartilaginous regeneration		
		(iv) Cartilage erosion		

**Table 4:** Summary of automated knee OA diagnosis and prognosis.

Task	Subtask	Area of OA management	Achievements	Future work suggestions	Machine learning techniques
Localization of knee joint	Detection of knee joint	Diagnosis	(i) Detected tibiofemoral joints on X-ray images [40]	(i) Recognition of OA features	(i) Histogram of oriented gradients [40–43]
			(ii) Detected patellofemoral joints on X-ray images [44]	(ii) Quantification of qualitative OA features	(ii) Local binary pattern [41, 42, 44]
					(iii) Random forest regression voting [44]
					(iv) Fully convolutional neural network [45, 46]
			(iii) Detected cartilage X-ray images [41, 42]		(v) YOLOv2 network [46]


	Segmentation of knee joint components	Diagnosis	(i) Segmented knee cartilage from 2D ultrasound images [27, 28]	(i) Area measurement	(i) Locally statistical level set method [28]
			(ii) Segmented knee cartilage from 2D MRI images [47]	(ii) Volumetric measurement	(ii) Automatic seed point detection [48]
			(iii) Segmented cartilage and meniscus from MRI images [29]	(iii) Joint shape measurement	(iii) Random walker [27]
			(iv) Segmented subchondral bone from multiple 2D MRI images [48]	(iv) Quantification of measurable OA features	(iv) Watershed
			(v) Segmented distal femur and proximal tibia from X-ray images [49]	(v) Reconstruction of 3D knee joint model for simulation and joint loading study	(v) Graph cut [27]
			(vi) Calculated joint space width on X-ray images [49]	(vi) Finite element analysis	(vi) Support vector machine classifier [43]
			(vii) Segmented femoral condyle cartilage from ultrasound images [50]	(vii) Utilization of statistical and computational models	(vii) Decision tree classifier [41, 42]
			(viii) Segmented bones (femur and tibia) and cartilages (femoral and tibial cartilages) on MRI images [51]		(viii) Active contour algorithm [42]
			(ix) Segmented knee bones, cartilage, and muscle tissues on MRI images [52, 53]		(ix) U-Net [29, 47, 54–57]
			(x) Segmented femoral cartilage and tibial cartilage from 3D MRI images [54, 58]		(x) Res-U-Net [49]
					(xi) Siam-U-Net [50]
					(xii) CUMed-Vision [49]
					(xiii) DeepLabv3 [49]
					(xiv) FC-DenseNet [47]
					(xv) LinkNet [47]
					(xvi) TernausNet [47]
					(xvii) AlbuNet [47]
					(xviii) Attention U-Net [47]
					(xix) LadderNet [47]
					(xx) Multi-atlas registration [51]
					(xxi) CycleGAN [51]
					(xxii) cGANs [52]
					(xxiii) Connected conditional random field model [53]
					(xxiv) Convolutional encoder-decoder model [53]

Classification of knee OA severity	N/A	Diagnosis	(i) Discriminated osteoarthritic knee based on MRI features [59]	(i) Risk stratification	(i) 3D-CNN [56]
			(ii) Discriminated patellofemoral OA based on X-ray images [44]	(ii) Classification of OA features	(ii) Deep Siamese CNN [60]
			(iii) Classified meniscal lesion using MRI data [56]	(iii) Classification of OA severity based on computational outcomes	(iii) CNN with LBP [40]
			(iv) Graded knee OA severity using X-ray images based on KL classification [40, 46, 60]		(iv) CNN with HOG [40]
					(v) ResNet [46, 61]
					(vi) VGG [46, 61]
					(vii) DenseNet [46, 55, 61, 62]
					(viii) InceptionV3 [46]
					(ix) GooLeNet [61]
					(x) ResNeXt [61]
					(xi) MobileNetV2 [61]
					(xii) Linear mixed-effects models [45]
					(xiii) Elastic net [45]
					(xiv) Support vector [59] machine [40]
					(xv) Random forest model [45, 56]
					(xvi) *K*-nearest neighbour [42]
					(xvii) Ensemble method using SE-ResNet-50 and SE-ResNet-50-32x4d [63]

Prediction of knee OA disease progression	Without intervention	Prognosis	(i) Estimated future knee OA incidence	(i) Risk stratification	(i) Random forest classifier [64, 65]
			(a) 30 months [64]	(ii) Selection of data from suitable time points to indicate short-term and long-term OA changes	(ii) Logistic regression classifier [66–69]
			(b) 48 months [70]	(iii) OA feature change detection	(iii) Support vector machine classifier [66]
			(c) 8 years	(iv) Discovery of pain-associated imaging features	(iv) XGBoost model [49]
			(ii) Predicted medial JSN progression [66]		(v) Multilayer perceptron [67, 71]
			(iii) Predicted radiographic joint space loss progression [67]		(vi) LASSO regression [39]
			(iv) Predicted knee OA onset and knee OA deterioration [71]		(vii) Artificial neural network [70]
			(v) Discriminated between progressors and nonprogressors [72]		(viii) Deep CNN [44, 72, 73]
			(vi) Predicted pain [73, 74]		(ix) DenseNet CNN [68]
			(vii) Predicted risk of progressive pain and structural change [65]		(x) Gradient boosting machine [44, 70]
			(viii) Predicted total knee replacement (TKR) incidence [68, 75]		(xi) Duo classifier [65]
					(xii) DeepSurv [75]
					(xiii) Dynamic functional mixed-effects model [54]

## Data Availability

All the data are included in the list of references.
